The article "Interfering with the Expression of Ubiquitin-Like with PHD and Ring Finger Domains 1 Can Inhibit the Invasion of Human Renal Cell Carcinoma" was retracted in 2023. Reasons: unreliable results or conclusions; concerns about the data; concerns about the peer review; concerns about the citations.

# Interfering with the Expression of Ubiquitin-Like with PHD and Ring Finger Domains 1 Can Inhibit the Invasion of Human Renal Cell Carcinoma

**DOI:** 10.1155/2022/6971131

**Published:** 2022-05-18

**Authors:** Susu Wu, Xiao Pan, Yanqun Cai, Caiqin Li

**Affiliations:** Department of Laboratory, Taizhou Municipal Hospital, No. 381-1, Zhongshan East Road, Jiaojiang District, Taizhou City 318000, China

## Abstract

**Objective:**

The ubiquitin-like with PHD and ring finger domains 1 (UHRF1) is a protein coding gene which is associated with colorectal cancer and other diseases. Therefore, the present study was aimed at investigating the effect and mechanism of UHRF1 protein on invasion and metastasis in human renal carcinoma cells.

**Methods:**

After UHRF1 was interfered with or overexpressed in renal carcinoma cell lines A498 and 769-P, the relative mRNA and protein level of UHRF1 was detected by RT-qPCR and immunofluorescence. The colony formation assay and MTT were performed to observe the proliferation and cell viability in each group. In addition, the invasion and metastasis of the cells in each group were detected by Transwell and wound healing assay. Finally, Western blot was utilized to measure protein expression of MMP-2 and MMP-9 and the level of protein in the Wnt/*β*-catenin signaling pathway.

**Results:**

The cell ability, proliferation, invasion, and metastasis in A498 and 769-P cells were inhibited after interfering with UHRF1. In addition, the expression of MMP-2, MMP-9, c-myc, and *β*-catenin was significantly decreased, while the expression of GSK-3*β* was significantly increased. However, contrasting results were demonstrated when UHRF1 was overexpressed.

**Conclusions:**

Interference with the expression of UHRF1 was able to inhibit the invasion and metastasis of human renal carcinoma cell lines A498 and 769-P, which may be related to mediating the Wnt/*β*-catenin signaling pathway and regulating the expression of MMP-2 and MMP-9.

## 1. Introduction

Renal cell carcinoma (RCC), which accounts for about 2%-3% of all malignancies, has taken the second incidence in China among malignancies of the urinary system, and the incidence has been increasing [1]. With the insidious onset, RCC has no specific symptoms in the early stage. As a result, when patients present with the typical triad signs of “hematuria, lumbodynia, and abdominal mass,” the tumor has broken through the renal collective system, infiltrated into the surrounding tissues, and even metastasized to distant tissues [2, 3]. At present, treatment for RCC is becoming increasingly mature, and surgical treatment for early tumors is effective. However, radiotherapy combined with chemotherapy or immunotherapy for tumors that have developed local or distant metastasis does not receive a satisfactory curative effect. What is worse, it is highly possible to arise tumor recurrence and metastasis after surgery without effective preventive measures. In recent years, metastatic RCC can be also treated with cytokine therapy or targeted drugs; however, the evaluation effect is still unsatisfactory in improving the objective response rate of patients as well as prolonging progression-free survival (PFS) and overall survival time (OS) [4]. Therefore, it is of great importance to study the invasion and metastasis mechanism of RCC at the molecular level.

Tumor invasion and metastasis is a complex biological process [5]. Gene regulation plays a crucial role in many processes, such as unlimited growth potential, epithelial-mesenchymal transition (EMT), and apoptosis avoidance [6]. The Wnt cell signaling pathway is one of the essential signaling pathways affecting the migration and invasion ability of cancer cells. When the Wnt/*β*-catenin cell signal transduction pathway is activated, Wnt secretes proteins to penetrate the cell membrane, which is aimed at degrading the GSK3*β*/APC/Axin/CKIa complex. Consequently, this process prevents *β*-catenin from being phosphorylated by the complex and gradually leads to *β*-catenin accumulation in the cytoplasm. When *β*-catenin is accumulated at a certain amount, it transfers to the nucleus and binds to the transcription T cell factor (TCF)/lymphoid enhancer-binding factor (LEF) to form a transcriptional complex. This complex subsequently activates its downstream target genes matrix metalloproteinases (MMPs), p21, and c-myc [7, 8]. Moreover, the overexpression of UHRF1 has been identified as a possible biomarker in a variety of malignancies, resulting in either DNA hypermethylation or global DNA hypomethylation, both of which contribute to cancer development, progression, and invasion [9]. MMPs are a group of proteolytic enzymes which are highly homologous and zinc-dependent. In the meanwhile, MMPs can degrade extracellular matrix components into small pores by breaking them down, so that tumor cells can spread through these pores and promote tumor invasion and metastasis [10]. In addition, the accumulation of *β*-catenin will enhance the interaction between N-cadherin and the cytoskeleton, thereby increasing its affinity to mesenchymal cells, which results in the invasion and metastasis of cancer cells [11].

Ubiquitin-like with PHD and ring finger domains 1 (UHRF1), a member of the UHRF family, is highly expressed in a variety of tumor tissues. Many studies have shown that UHRF1 is closely related to different kinds of cell proliferation, invasion, and metastasis. In addition, Daskalos et al. [12] found that UHRF1 in lung cancer cells induces tumor suppressor genes RASSF1, CYGB, and CDH13 promoter methylation. By inhibiting their expression, UHRF1 can promote tumor cell invasion. Moreover, Zhou et al. [13] pointed out that UHRF1 promotes the promoter methylation of Slit3, CDH4, and RUNX3, thereby accelerating the invasion and metastasis of gastric cancer cells. UHRF1 in hepatocellular carcinoma may strengthen the invasive characteristics through the regulation of genomic stability and p53, thereby boosting tumor progression [14]. From this, it can be obtained that in different tumor types, UHRF1 regulates the expression of tumor suppressor genes via different genetic mechanisms, which influence the invasion and migration of cancer cells. Adding to that, Wang et al.'s in vitro assay has confirmed that UHRF1 is highly expressed in renal cancer tissues [15]. By interfering with its expression, the proliferation, migration, and invasion of renal cancer cells are hoped to be inhibited. However, the specific regulatory mechanism of UHRF1 is still unclear. Therefore, this study is aimed at investigating the mechanism of UHRF1 on the invasion and metastasis of renal carcinoma cells. The research results will provide more effective guidance and assistance for the diagnosis, treatment, and prognosis evaluation of RCC in the future.

## 2. Materials and Methods

### 2.1. Cell Culture and Cell Transfection

Human renal epithelial cell (HK-2), human renal cancer cell line A498, Caki-1, and 769-P were purchased from Shanghai Cell Bank (Shanghai, China). HK-2 was cultured in DMEM/F-12, 769-P and A498 cells were cultured in RPMI-1640 medium, and Caki-1 was cultured in McCoy's 5A medium (Gibco, USA), which contained 10% fetal bovine serum (FBS, Gibco). The medium was put in a saturated humidity incubator at 37°C with 5% CO_2_.

siRNA (si-UHRF1) against UHRF1 and negative control (Si-NC) were designed and synthesized by Ruibo Biotechnology Co., Ltd (Guangzhou, China). Overexpressing plasmid pcDNA3.1-UHRF1 (UHRF1) in UHRF1 along with control vector (vector) were purchased from General Biol (Anhui, China). A498 was cultured in 6-well plates. Six groups, namely, blank group (blank), si-UHRF1 group, si-NC, UHRF1, and vector, were established. In line with the manufacturer's instructions, all cell transfections were performed using Lipofectamine 2000 (Invitrogen, CA, USA).

### 2.2. Reason for Selecting Cell Lines A498 and 769-P

The cell lines A498 and 769-P were established which harbor mutated and secrete high levels of vascular endothelial growth factor (VEGF). These cell lines have high tumorigenicity that may enhance the tumor formation even after serial passage in naked mice retaining their original histological characters.

### 2.3. MTT Assay

The cell proliferation in each group was observed by the MTT assay (Gibco, USA). After cells in each group were transfected for 48 hours, 769-P and A498 cells were plated into 96-well plates (6000 cells/well) and incubated for 1, 2, and 3 days. Then, 20 *μ*l MTT (5 mg/ml; Gibco, USA) was added to each well and cultured for 4 h. Subsequently, the culture medium was removed, and 150 *μ*l DMSO was used to dissolve the crystals. The absorbance was measured at 570 nm using a microplate reader.

### 2.4. Immunofluorescence Assay

After cells in each group were transfected for 48 hours, they were fixed with 4% paraformaldehyde for 15 minutes. Subsequently, cells with 0.5% Triton X-100 were continually cultured for 20 minutes at room temperature. Afterward, excess liquid was aspirated, and cells were blocked with goat serum. 30 minutes later, UHRF1 primary antibody solution (ab57083, Abcam) was added and incubated overnight at 4°C. Fluorescent secondary antibody anti-LPO antibody (HRP) was added the next day and incubated for 1 hour at 37°C. After that, the samples were incubated with DAPI in the dark for 5 minutes. Nuclei were then stained and rinsed four times using PBST. After the excess liquid was aspirated, a mounting solution containing antifluorescent quenchant was utilized to mount the samples whose images were observed and collected under a fluorescence microscope.

### 2.5. Colony Formation Assay

The viability of cells in each group was observed via the colony formation assay. The cells in each group were rinsed twice with PBS. Afterward, individual cells in each group were obtained with 0.25% trypsin and then inoculated into culture dishes for one hour. Serially dilute the samples to obtain 100 cells in a 10 ml culture medium. At last, the cells were inoculated into other culture dishes for 10-14 days, followed by an observation of the cell colony formation under a microscope.

### 2.6. Transwell Assay

The invasion ability of cells in each group was evaluated by the Transwell assay. After the Transwell chamber was prepared, ECM gel was paved in the upper chamber, while a medium containing 10% serum was added to the lower chamber and allowed to stand for 4 hours. After that, cells in each group were seeded in the upper chamber, respectively, and cultured for 24 hours. Then, they were taken out, fixed in ethanol, and stained with crystal violet solution. Finally, cell invasion was observed under a microscope (×100).

### 2.7. Wound Healing Assay

A498 and 769-P cells were cultures in 6-well plates (1 × 10^5^ cells/well); after 48 h of transfection, a 200 *μ*l pipette tip was used to form linear scratches on the cell monolayer. Then, the cells were cultured in a 5% CO_2_ incubator at 37°C under standard conditions. After the image of the wound was taken by a microscope (Nikon Corporation), the width of the wound was calculated using ImageJ software.

### 2.8. RT-qPCR Assay

Total RNA in each group was extracted by TRIzol. Afterward, RNA was reversely transcribed into cDNA after passing the RNA purity and integrity tests. Subsequently, RT-qPCR assays were performed with reaction conditions: 96°C for 4 minutes, 94°C for 30 seconds, 58°C for 30 seconds, and 72°C for 30 seconds, repeat 40 times. The relative expression of mRNA was assessed with the 2^−∆∆Ct^ method, with GAPDH as an internal reference. Primer sequences are displayed in Table 1.

### 2.9. Western Blot

When total cellular protein from each group was extracted, the protein concentration was determined using a BCA protein quantification kit (Pierce, 23225). Proteins were separated with 12% SDS-PAGE and transferred to PVDF membranes. After blocking with 5% skim milk powder at room temperature, the membranes were incubated overnight at 4°C with primary antibody MMP-9 (1 : 1000 dilution, ab58803, Abcam), MMP-2 (1 : 1000 dilution, ab92536, Abcam), *β*-catenin (1 : 1000 dilution, ab16051, Abcam), GSK-3*β* (1 : 1000 dilution, ab93926, Abcam), c-myc (1 : 1000 dilution, ab32072, Abcam), and *β*-actin (1 : 800 dilution, ab179467, Abcam). The next day, the membranes were washed three times with PBS and incubated with the secondary antibody goat anti-rabbit IgG-HRP (1 : 1500 dilution, Bioworld Company) for 90 minutes at room temperature. Finally, the ECL chromogenic substrate was added for color reaction. The results were analyzed by ImageJ software.

### 2.10. Statistical Analysis

The experimental data were expressed as the mean ± standard deviation (SD), and SPSS 21.0 software was utilized for statistical analysis. In addition, the *t*-test method was used for comparison between the two groups. *p* < 0.05 was considered that the results were statistically significant.

## 3. Results

### 3.1. UHRF1 Is Highly Expressed in Renal Carcinoma Cells

To examine the effect of UHRF1 expression on the function of renal cancer cells, we compared the expression of UHRF1 in normal renal cells and renal carcinoma cells and found that UHRF1 was significantly upregulated in renal carcinoma cells than normal renal cells (HK-2) and was highly expressed in A498 and 769-P cells (Figure 1(a)). UHRF1 siRNA (si-UHRF1) or overexpressing plasmid (Pc-UHRF1) in A498 cells was transfected to downregulate or upregulate UHRF1 expression. Knockout of UHRF1 can inhibit its expression in A498 and 769-P cells, while overexpression can reverse the result (Figures 1(b) and 1(c)), which indicate that transfection is successful. The results of the immunofluorescence assay (Figures 1(d) and 1(e)) showed that UHRF1 was mainly expressed in the nucleus of A498 and 769-P cells. Compared with the si-NC group, the expression of UHRF1 in the si-UHRF1 group was decreased. However, compared with the vector group, the expression of UHRF1 in the UHRF1 group was increased. The results indicated that UHRF1 is highly expressed in renal carcinoma cells.

### 3.2. Inhibition of UHRF1 Can Inhibit the Proliferation and Cell Viability of Renal Carcinoma Cells

Cell proliferation was further examined by the MTT assay. The results (Figures 2(a) and 2(b)) confirmed that the ability of proliferation of A498 and 769-P cells in the si-UHRF1 group was significantly reduced compared with the si-NC group. On the contrary, the ability of A498 and 769-P cells in the UHRF1 group was significantly increased compared with the vector group. A colony formation assay was utilized to evaluate the cell viability of A498 and 769-P cells (Figure 2(c)). We found that knockout of UHRF1 can inhibit the cell viability of A498 and 769-P cells, and overexpression of UHRF1 can significantly motivate it. The results showed that UHRF1 was involved in the proliferation and cell viability of renal cancer cells.

### 3.3. Inhibition of UHRF1 Can Inhibit Invasion and Metastasis of Renal Carcinoma Cells

Further, we examined the effects of UHRF1 on invasion and metastasis in renal carcinoma cells. Transwell and wound healing assays were, respectively, utilized to evaluate the invasive and metastasizing ability of A498 and 769-P cells. The results (Figures 3(a) and 3(b)) suggested that the invasion and metastasis of A498 and 769-P cells were significantly decreased after interfering with UHRF1 expression compared with the si-NC group. Instead, the invasion and metastasis of A498 and 769-P cells were significantly increased after overexpressing UHRF1 compared with the vector group (*p* < 0.05). To further investigate the mechanism by which UHRF1 regulates functional changes in renal cancer cells, the levels of MMP-2 and MMP-9 were examined, which are closely related to the invasion and metastasis of tumor cells (Figure 3(c)). It showed that the expression of MMP-2 and MMP-9 in A498 and 769-P cells was significantly increased after interfering with UHRF1 expression. However, the expression of MMP-2 and MMP-9 significantly decreased after overexpressing UHRF1.

### 3.4. Inhibition of UHRF1 Can Inhibit the Expression Levels of Wnt/*β*-Catenin Signaling Proteins

The effect of UHRF1 expression on the Wnt/*β*-catenin signaling pathway which associates with tumor metastasis was detected. Western blot indicated (Figure 4) that the expression levels of *β*-catenin and c-myc in A498 and 769-P cells in the si-UHRF1 group were significantly decreased; while the expression levels of GSK-3*β* were increased compared with the si-UHRF1 group. These results confirmed that the activation of the Wnt/*β*-catenin signaling pathway was inhibited after interfering with the expression of UHRF1.

## 4. Discussion

As the most common renal malignant tumor with insidious onset and strong invasiveness in clinical practice, RCC is mostly found in the late stage when radiotherapy, chemotherapy, and other treatments are not effective. However, surgery in the early stage is currently the most effective treatment [16]. Consequently, it has become one of the research focus in exploring the molecular mechanism of malignant growth and metastasis to provide new treatment strategies for RCC. UHRF1, as an important epigenomic regulator, is involved in tumor development [17, 18]. In the present study, we compared the expression of UHRF1 in normal renal cells and renal carcinoma cells to see if it influenced renal cancer cell function. We found that UHRF1 was significantly upregulated in renal carcinoma cells compared to normal renal cells (HK-2) and was overexpressed in A498 and 769-P cells as given in Figure 1(a). In contrast, a study conducted by Achour et al. found and concluded that the downregulation of UHRF1 is dependent upon the generation of reactive oxygen species (ROS) [19]. However, the downregulation of UHRF1 could significantly express the tumor suppressor genes [20]. Previously, many studies have confirmed that UHRF1 can be used as a molecular marker for cancer diagnosis and prognosis [21–23]. For instance, Hu et al. demonstrated that UHRF1 might be able to promote the proliferation of pancreatic cancer by inhibiting SIRT4 [24]. Lee et al. found that interfering with UHRF1 could lead to the death of early cervical cancer cells. Although it has been found that upregulation of UHRF1 can promote metastasis and poor prognosis of RCC, the mechanism by which UHRF1 regulates RCC is not clear [25].

The Wnt signal is divided into the typical Wnt pathway and two atypical Wnt pathways [26]. The typical Wnt signaling pathway (namely, the Wnt/*β*-catenin signaling pathway) is currently the most widely studied in clinical practice. Studies have demonstrated that nearly 50% of currently known tumors show an association with abnormal regulation of the Wnt/*β*-catenin signaling pathway, such as intestinal cancer [27] and breast cancer [28, 29]. Abnormal expression of proteins such as GSK-3*β* [30], *β*-catenin [3], and MMPs [10] in the pathway triggers sustained cell proliferation, ultimately leading to cancer [31]. The scaffold protein Axin coordinates a dual-kinase process that phosphorylates the N-terminus of cytosolic *β*-catenin. *β*-catenin, CK1, GSK3, and other components necessary for Wnt-dependent signaling events have binding sites on Axin. CK1 family members phosphorylate *β*-catenin at serine 45. This priming phosphorylation is essential for GSK3 to phosphorylate residues 41, 37, and 33 in the future [32]. In the meanwhile, it plays a crucial role in the invasion and metastasis of cancer cells [33, 34]. Therefore, the present study investigated whether UHRF1 could mediate the invasion and metastasis of renal cancer cells by regulating the Wnt/*β*-catenin signaling pathway.

In the present study, proliferation and invasion of A498 and 769-P renal cancer cells were reduced after interfering with UHRF1 expression. However, the proliferative and invasive capacity of cells increased after overexpressing UHRF1, having confirmed that UHRF1 was involved in the progression of RCC. In addition, Western blot showed that the expression of MMP-2, MMP-9, c-myc, and *β*-catenin was decreased, while the expression of GSK-3*β* was increased in A498 and 769-P renal cancer cells after interfering with UHRF1 expression. However, the opposite results were presented after overexpression of UHRF1. These findings suggest that downregulation of UHRF1 can inhibit the Wnt/*β*-catenin signaling pathway and gradually inhibit invasion and metastasis of A498 and 769-P cells. The UHRF1 was found to be the promoter of *β*-catenin; however, for development and carcinogenesis, Wnt regulation of *β*-catenin degradation is critical. Glycogen synthase kinase-3 (GSK-3) in association with tumor suppressor proteins Axin and adenomatous polyposis coli is thought to begin *β*-catenin breakdown at the amino-terminal serine/threonine phosphorylation (APC) [35].

## 5. Conclusion

The functional and modulation processes of the UHRF1 protein complex have advanced significantly, and it is anticipated to become a universal biomarker for cancer and a specific target for cancer therapy. By interfering with UHRF1 expression, invasion and metastasis of renal cancer cells A498 and 769-P could be inhibited. This result could be obtained by mediating the Wnt/*β*-catenin signaling pathway. This study provides a more comprehensive theoretical basis for UHRF1 as a therapeutic target in patients with RCC.

## Figures and Tables

**Figure 1:** The expression of UHRF1 in A498 and 769-P cells: (a) the expression of UHRF1 in normal renal cells and renal carcinoma cells detected by RT-qPCR, ^∗^*p* < 0.05 and ^∗∗^*p* < 0.01*vs.* HK-2; (b) the expression of UHRF1 in A498 cells detected by RT-qPCR, ^∗∗^*p* < 0.01*vs.* si-NC, ^##^*p* < 0.01*vs.* vector; (c) the expression of UHRF1 in 769-P cells detected by RT-qPCR, ^∗∗^*p* < 0.01*vs.* si-NC, ^##^*p* < 0.01*vs.* vector; (d) UHRF1 expression in A498 cells detected by immunofluorescence assay; (e) UHRF1 expression in 769-P cells detected by immunofluorescence assay.

**Figure 2:** Effect of UHRF1 expression on proliferation and cell viability of renal carcinoma cells: (a) cell proliferation of A498 cells detected by MTT; (b) cell proliferation of 769-P cells detected by MTT; (c) cell viability of A498 and 769-P cells detected by colony formation assay: ^∗∗^*p* < 0.01*vs.* si-NC group; ^#^*p* < 0.05 and ^##^*p* < 0.01*vs.* vector group.

**Figure 3:** Effect of UHRF1 expression on invasion and metastasis of renal carcinoma cells: (a) effect of UHRF1 expression on invasive ability of A498 and 769-P cells detected by Transwell; (b) effect of UHRF1 expression on metastasizing ability of A498 and 769-P cells detected by wound healing assay: ^∗∗^*p* < 0.01*vs.* si-NC group; ^##^*p* < 0.01*vs.* vector group.

**Figure 4:** Effect of UHRF1 expression on Wnt/*β*-catenin signaling pathway. ^∗∗^*p* < 0.01*vs.* si-NC group; ^##^*p* < 0.01*vs.* vector group.

**Table 1:** Primer sequences.

Gene	Forward primer	Reverse primer
UHRF1	5′-ACTTGGAGGCCTTGGCTAAC-3′	5′-GACAGACAGACTGCGACCTG-3′
GAPDH	5′-TGTGTCCGTCGTGGATCTGA-3′	5′-TTGCTGTTGAAGTCGCAGGAG-3′

## Data Availability

The data used to support the findings of this study are available from the corresponding author upon request.
